# The Clinical Diagnostic Value of Lumbar Intervertebral Disc Herniation Based on MRI Images

This article has been retracted.

**DOI:** 10.1155/2021/5594920

**Published:** 2021-04-05

**Authors:** Kangxing Zheng, Zihuan Wen, Dehuai Li

**Affiliations:** ^1^Shangrao Municipal Hospital, Shangrao, Jiangxi 334000, China; ^2^Harbin Second Hospital, Harbin, Heilongjiang 150056, China

## Abstract

MRI was used to measure the changes in the angle of the facet joints of the lumbar spine and analyze the relationship between it and the herniated lumbar intervertebral disc. Analysis of the causes of lumbar disc herniation from the anatomy and morphology of the spine provides a basis for the early diagnosis and prevention of lumbar disc herniation. There is a certain correlation between the changes shown in MRI imaging of lumbar disc herniation and the TCM syndromes of lumbar intervertebral disc herniation. There is a correlation between the syndromes of lumbar disc herniation and the direct signs of MRI: pathological type, herniated position, and degree of herniation. Indirect signs with MR, nerve root compression and dural sac compression, are related. The MRI examination results can help syndrome differentiation to improve its accuracy to a certain extent. MRI has high sensitivity for the measurement of the angle of the facet joints of the lumbar spine and can be used to study the correlation between the changes of the facet joint angles and the herniated disc. Facet joint asymmetry is closely related to lateral lumbar disc herniation, which may be one of its pathogenesis factors. The herniated intervertebral disc is mostly on the sagittal side of the facet joint, and the facet joint angle on the side of the herniated disc is more sagittal. The asymmetry of the facet joints is not related to the central lumbar disc herniation, and the angle of the facet joints on both sides of the central lumbar disc herniation is partial sagittal.

## 1. Introduction

Lumbar intervertebral disc herniation refers to the rupture of the annulus fibrosus due to various reasons such as lumbar degeneration and chronic strain. The nucleus pulposus moves laterally or backwards, protruding very laterally or directly behind the ruptured annulus [1]. The low back pain caused by stimulation of the spinal nerve root and cauda equina is accompanied by localized radiating pain and numbness of the lower limbs or even a clinical syndrome of fecal dysfunction or decreased muscle strength of the lower limbs. Because of its long course of disease, easy recurrence, and complicated conditions, it seriously affects the life and work of patients. With the development of modern medicine, people gradually deepen their understanding of the disease.

In today's society, the incidence of lower back and leg pain is increasing, and the age and severity trend are increasing, which has caused a huge burden and pressure on society, and has gradually become one of the main diseases threatening human health. Lumbar facet joints (LFJ) degeneration, lumber disc herniation (LDH) stimulation, or compression of the corresponding segmental nerve roots are among the causes of low back pain. Whether the structural abnormality of the functional unit of the spine caused by LFJ degeneration causes the abnormal force of the lumbar intervertebral disc herniation is unclear, and whether lumbar facet joint angle changes are common in patients with lumbar disc herniation is still unclear [2]. A full understanding of the relationship between lumbar facet joint angle changes and lumbar disc herniation is helpful to the prevention and treatment of low back pain. The lumbar spine is the structure with the largest range of motion and weight-bearing in the lower part of the spine. The intervertebral disc and the posterior facet joint (FJ) constitute the “three-joint complex,” which bears the weight of the function of spinal unfit (FSU) and plays an important role in activities in all directions [3]. A large number of studies have shown that there is a close relationship between facet joint angle changes and intervertebral disc herniation, and the two influence each other in the occurrence and development of the entire lumbar degenerative disease. Lumbar disc herniation is defined as a pathological condition caused by focal displacement of the nucleus pulposus, annulus, or endplate in the lumbar intervertebral disc that exceeds the normal peripheral boundary of the intervertebral disc, compressing the corresponding segment of the dural sac or nerve root [4]. At present, the general definition of intervertebral disc herniation in clinical medicine is rather confusing. There are both intraoperative pathological classification and imaging data evaluation classification. The evaluation methods are diverse, but there is no uniform standard. Some papers equate intervertebral disc protrusion with intervertebral disc herniation, that is, the limited intervertebral disc tissue (nucleus pulposus, part of the annulus fibrosus) protrudes into the spinal canal through the posterior annulus fibrosus, and the posterior longitudinal ligament ends ruptured [5].

In this study, the MRI images showing prolapsed and free intervertebral discs are also included in the scope of intervertebral disc herniation. According to Wiltse's classification method, referring to related works, it is divided into four areas, namely, the central area of the spinal canal, the subarticular joint area, the foramen area, and the foramen area [6] You can refer to related works to locate the intervertebral disc herniation. The morphological classification of herniated discs in MRI imaging is summarized as follows. Central type: intervertebral disc tissues (nucleus pulposus, part of annulus fibrosus) protrude posteriorly into the central canal area through the posterior longitudinal ligament, compressing the dural sac and (or) two lateral nerve roots, causing partial stenosis of the central spinal canal [7]. Paracentral type: intervertebral disc tissue (nucleus pulposus, part of annulus fibrosis) passes through the posterior longitudinal ligament and enters the subarticular area and (or) one side of the central spinal canal through the posterior longitudinal ligament. Part of the dural sac and the nerve root on the same side are compressed, and part of the central spinal canal and lateral recesses on this side are narrowed [8]. Lateral type: the intervertebral disc tissue (nucleus pulposus, part of annulus fibrosis) protrudes back into the intervertebral foramen area through one posterior longitudinal ligament, compressing the nerve root, and the lateral recess can be narrowed. Extremely lateral type: the disc group (nucleus pulposus, part of the annulus fibrosus) protrudes into the outer foramen area or outside of the nerve root exit area, compressing the upper segment of the nerve root. In order to facilitate the study, we combined the paracentral type and lateral type into the lateral LDH group in the study.

## 2. Signs of Lumbar Disc Herniation in MRI Diagnosis

Lumbar disc herniation refers to the partial or complete rupture of the lumbar intervertebral disc fibrous annulus due to various reasons such as degeneration, strain, and injury, and the nucleus pulposus tissue protrudes backward or to one side from the rupture or even irritates or compresses the dura mater and then oppresses the lumbar spinal nerve roots and cauda equina, causing low back pain with radiating pain in the legs and even bladder muscle and rectal dysfunction, which are manifested by clinical symptoms such as poor urination and defecation [8]. It is a common clinical disease and frequently occurring disease. In the early stage, patients mostly complained of low back pain. In the later stage, the main complaints are leg pain and radiating pain. In severe cases, it will be disabled and the quality of life of the patient will be severe, and it will bring a great economic burden to the society. This has become a major public health issue. Therefore, the treatment effect of lumbar intervertebral disc herniation is particularly important. The premise of treatment is diagnosis [9]. The essence of TCM syndrome differentiation guides clinical legislation and prescriptions. Correct syndrome differentiation is directly related to treatment methods. Therefore, combining modern medicine to make TCM syndrome differentiation more standardized and scientific is TCM. Schematic of magnetic resonance imaging is shown in Figure 1.

### 2.1. Advantages of MRI in the Diagnosis of Lumbar Disc Herniation

The biggest advantage of magnetic resonance imaging is that it can obtain images through horizontal and sagittal three-dimensional scanning, different sequences, and imaging techniques and directly observe the normality of the spinal cord, subarachnoid space, vertebral body, and intervertebral discs. For intervertebral disc disease, the signal level can be directly observed. There is a relationship between the position, direction, shape, and size of the nucleus pulposus and the nerve roots of intervertebral disc herniation. Prolapse and free types are also acceptable which show the relationship with the original intervertebral disc [10]. Compared with traditional imaging methods, it has obvious advantages. Scholars have found that, in the diagnosis of lumbar disc herniation, myelography is not as sensitive as MRI, and MRI has a higher positive rate [11]. Compared with CT, it has more imaging parameters, multiple tissue variable functions, more flexible and extensive, no radiation, and no damage to the human body, and its diagnostic accuracy is better than that of CT scan.

Using the American GE 1.5THDE MRI machine, the sagittal image adopts T1-weighted phase and T2-weighted phase, and the cross-sectional image adopts T2-weighted phase image. The line of the image is parallel to the lumbar vertebral body endplate, up to the lower end of the upper vertebral body Plate, down to the upper endplate of the lower vertebral body, is protruding the intervertebral disc tissue upward or downward to extend the scanning range. The images of each layer are separated by 1-2 mm, and 4-5 cross sections of each intervertebral space are taken from top to bottom, and the L3/4, L4/5, and L5/S1 intervertebral spaces are scanned. And, save all the image data to the image processing workstation of the imaging department for registration and archive. The shape of the herniated disc in the MRI image is shown in Figure 2.

### 2.2. Direct Signs of Lumbar Disc Herniation

#### 2.2.1. Prominence of Nucleus Pulposus

Herniated intervertebral disc, on the sagittal plane, on the proton density image or T2-weighted image, is hemispherical or tongue-like with moderately high signal. Outside the low-signal fibrous ring, it is the backward (central type) or laterally posterior (lateral posterior) type; the signal intensity of the tissue is equal to that of the degenerated intervertebral disc, higher than the cerebrospinal fluid signal, and lower than the epidural fat signal; on the T1-weighted image, the signal intensity is often the same as that of the central part of the nondegenerated intervertebral disc [12]. In the same, high, or low signal, the signal intensity is lower than the cerebrospinal fluid, higher than the spinal cord, and slightly lower or higher than the extradural fat; at the degeneration of the intervertebral disc, the signal varies according to the degree of degeneration of the nucleus pulposus, the nucleus pulposus herniated and not. There is a “narrow neck” connected between the protrusions.

#### 2.2.2. Free Nucleus Pulposus

A large piece of nucleus pulposus tissue penetrates the annulus fibrosus and posterior longitudinal ligament, completely protrudes into the spinal canal, and is separated from the original disc. Free fragments of the nucleus pulposus can be seen free in the spinal canal or even in the subarachnoid space of the dura, compressing the cauda equina nerve or nerve root. On the sagittal plane, it is easier to show the free intervertebral disc on the level of the diseased intervertebral disc or in the lower spinal canal.

#### 2.2.3. Schmorl Nodules

It appears as a semicircular or square impression on the upper or lower edge of the vertebral body. The content and the same level of the nucleus pulposus and other signals can be seen on the T1-weighted image of the MRI examination [13, 14]. There is a thin low-signal zone around the vertebral body, which is the cartilage plate of the vertebral body. Rupture is a special disc herniation in which the nucleus pulposus protrudes into the cancellous bone of the vertebra through the fissure.

#### 2.2.4. Herniated Degree of Intervertebral Disc

By measuring the cross-sectional image of the magnetic resonance examination of patients with lumbar disc herniation, the distance between the herniated disc and the herniated disc in the cross-section is analyzed, and the degree of herniation is divided into three degrees of light, medium, and severe, and the degree of vertebral body protrusion is less than 0.3 cm for mild, the degree of vertebral body protrusion is moderate between 0.3 cm and 0.5 cm, and the degree of vertebral body protrusion greater than 0.5 cm is severe [15].

### 2.3. Indirect Signs of Lumbar Disc Herniation

#### 2.3.1. Lumbar Dural Sac Compression

The dural sac refers to a sac-like structure composed of the dura mater. The place where nerves converge is a tissue that protects the spinal cord. When the intervertebral disc is herniated, the dural sac will be deformed by pressure, and the intervertebral disc and its interdural fat will be displaced [16]. When the herniation is large, the dural sac will be significantly deformed, and its crescent-shaped fissure will shrink. The dural space change can be seen on the MRI image.

#### 2.3.2. The Nerve Roots of the Lumbar Spine Are Compressed

The lumbar nerve root from leaving the dural sac to the outer mouth of the intervertebral canal can be divided into two segments: the nerve root canal and the intervertebral canal, passing through the disc yellow space, superior paraarticular groove, lateral recess, and pedicle physiological narrow passages such as inferior sulcus can stimulate or compress nerve roots and cause corresponding clinical symptoms. The MR imaging of nerve root compression caused by intervertebral disc herniation is closely related to the abnormal intervertebral disc signal shadow, which is closely related to the high signal nerve root. The nerve root is changed, and the nerve root is abnormally swollen and thickened.

#### 2.3.3. Lumbar Spinal Cord Compression

The compressed segment of the spinal cord shows abnormal signals of equal or long T1 and long T2, which are edema or ischemic changes in the spinal cord.

The causes of lumbar disc herniation include degenerative changes of the lumbar intervertebral disc, injury, weakness of the intervertebral disc's own anatomical factors, genetic factors, lumbosacral congenital abnormalities, and predisposing factors [11]. Degenerative changes of lumbar intervertebral discs: decreased water content of nucleus pulposus, and small-scale pathological changes such as instability and loosening of vertebral segments. Injury: slight damage caused by external force and aggravated degeneration. Weakness of intervertebral disc's own anatomical factors: human intervertebral disc blood circulation gradually lacks in adulthood, and its self-repair ability becomes worse. Genetic factors: there are reports of familial incidence of lumbar disc herniation [17]. Congenital abnormalities of the lumbosacral: sacralization of the lumbar spine, hemivertebral deformity, asymmetry of the articular process, etc., change the stress on the lower lumbar spine, which is prone to degeneration and injury. Inducing factors: factors such as increased abdominal pressure, waist posture, pregnancy, and other factors that can induce a sudden increase in intervertebral space pressure can cause nucleus pulposus herniation. The clinical classification is bulging type, prominent type, prolapsed free type, and Schmorl nodules. The clinical symptoms include low back pain, lower limb radiating pain, and cauda equina symptoms. The signs include lumbar scoliosis, restricted lumbar movement, tenderness, percussion pain, and sacral spinal spasm. Nuclear magnetic resonance was discovered by Bloch and Passel in 1946, so they won the Nobel Prize and carried out in-depth research on nuclear magnetic resonance [18]. MRI applies a certain frequency of radio frequency pulses to the human body in a static magnetic field so that the hydrogen protons in the human body are excited to cause magnetic resonance. After the pulse is stopped, the proton generates an MR signal during the relaxation process. MR signals are generated through processing procedures such as receiving, spatial coding, and image reconstruction of MR signals. Nerve root symptoms are a relatively prominent and common symptom in patients with lumbar disc herniation. As far as its pathogenesis is concerned, the current reasonable explanation is that mechanical compression causes neurological dysfunction, but it has not been excluded that the nerve root and nucleus pulposus contact. MRM uses multiple T2WI effects to suppress surrounding tissue signals and highlight static fluid-cerebrospinal fluid signals, thereby obtaining high-quality overall images of the subarachnoid space. Studies have shown that MRM can display nerve root compression well, and its ability is better than MRI. It has high application value for the exclusion and confirmation of the responsible intervertebral disc of PLID patients. The results of this study show that the combined use of MRI and MRM is more sensitive than conventional MRI. In summary, magnetic resonance imaging analysis of lumbar disc herniation has high diagnostic value.

## 3. MRI Study of Lumbar Disc Herniation

MR diagnosis of intervertebral disc herniation is significantly better than CT. It has a greater advantage than CT in imaging the structure of the spinal canal in the spine. The diagnostic rate of the degree of intervertebral disc degeneration, nerve root and dural compression, and spinal cord degeneration in LDH patients is significantly higher than that of CT. CT is in calcified intervertebral discs. It has advantages over MRI in the diagnosis of puff. High sensitivity to the morphology and signal changes of the compressed spinal cord so that MRI can effectively distinguish the morphology of the spinal cord with herniated nucleus pulposus, especially for the diagnosis rate of free nucleus pulposus in the differentiation of epidural masses and epidural masses. Smorgick et al. [15] studied the detection rate of MRI on the types of intervertebral disc herniation. The central herniation was 53.9%, the lateral herniation 29.7%, the foraminal type 12.5%, and the free type 4%. Magnetic resonance myelography (MRM) is slightly more sensitive than MRI in the diagnosis of the type of intervertebral disc herniation, but there is no significant difference in the consistency, accuracy, and specificity of the clinical diagnosis between the two. However, the disadvantage of MRM is that it needs to use a contrast agent and the operation is cumbersome. Compared with MRI, LDH is faster and more convenient. Cheung and Luk [16] reported that the accuracy of MRI in the diagnosis of intervertebral disc herniation is significantly higher than that of CT, and the accuracy of the diagnosis of intervertebral disc herniation and free intervertebral disc nucleus pulposus is 100%, which is significantly higher than that of CT examination of 88% and 50% LDH. The total detection rate of LDH by MRI is 96.67%, which is significantly higher than 71.67% of CT. For the diagnosis of lumbar facet joints in the comparison of CT and MRI, LewandrowskI et al. [17] believe that MRI is an indispensable tool. The evaluation accuracy of FJ degeneration degree is 94% of CT. Osteophyte hyperplasia, gas accumulation in facet joints, and vacuum phenomenon will affect the accuracy of articular cartilage thickness measurement. Raudner et al. [18] pointed out that although the sensitivity of FJ boundary measurement in the MRI sagittal image is not as good as that of CT scan, the clarity can fully meet the needs of measurement research. In this study, the cross-sectional images of the MRI were used to measure the angles of the articular processes on both sides. Some of the cases in the study included CT imaging data. In the study, we found that, according to the measurement method developed by Beulah et al. [19], the joint angle on the horizontal axis of MRI meets the requirements of sports. The clarity of the facet joint image can fully meet the measurement requirements. For the control of measurement errors, we use two spine surgeons to measure in a double-blind situation and take the average of the measurement results as the final data result. The images of the measured cases that are seriously degenerated and which have unclear FJ surface will be excluded. A total of 500 cases included in the study underwent CT and MRI examinations at the same time. The left and right facet joint angles of the L3/4, L4/5, and L5/S1 segments measured by MRI and CT were subjected to independent sample *T*-test. The *P* value >0.05 indicates that the FJ angle measured by the two imaging methods is not statistically significant. MRI is used to measure the lumbar facet joint angle with high sensitivity and can be used to measure the facet joint angle change and analyze its relationship with herniated disc [20].

### 3.1. Clinical Data

Select 500 hospitalized electronic medical records from January 2019 to December 2019 with a clinical diagnosis of lumbar disc herniation and concurrent lumbar disc MRI examination, including 227 males and 273 females, with an average age range of 18–85 years. The age is 41.25 ± 3.02 years old, the course of disease is between 1 day and 20 years, and the average course of disease is 10.41 ± 1.21 months.

### 3.2. MRI Diagnostic Criteria

1. Direct signs can be seen in the low signal outside the annulus T1 and other signals and T2 medium and long signals. In the case of obvious degeneration, T2 has short signals, and it can be seen that the intervertebral disc is thinning in the sagittal position, and the intervertebral disc in the transverse position exceeds the edge of the vertebral body. The nucleus is connected by a “narrow neck” to form the nucleus pulposus. If the protrusion is not connected with the nucleus pulposus, the nucleus pulposus is free. The free position and shape can be imaged at one time in the sagittal position, and the upper or lower edge of the vertebral body can be directly seen with the nucleus pulposus isometric semicircular or square-like Schmorl nodules (Schmorl nodules) [16].
2. Indirect signs can show compression of the dural sac, nerve root or spinal cord, compression and tortuous epidural venous plexus, and changes in the bone structure and bone marrow of the interphase zone.

### 3.3. Case Inclusion Criteria

1. Those who meet the above diagnostic criteria and syndrome differentiation criteria
2. Aged over 18 years old, no gender limit
3. Hospitalized cases with complete relevant imaging data and clinical case data
4. The imaging diagnosis report is completed by two or more imaging physicians

### 3.4. Scanning Method

Place the coil and fix it on the examination bed. The patient lies on its back, the long axis of the body is consistent with the long axis of the bed, and the arms are placed on both sides of the body or crossed in front of the chest and abdomen so that the patient's position is relaxed and suitable. The shoulders should be pushed up as far as possible so that the lower part of the joint coil can include the tail of the skeletal body, the sagittal positioning cursor is directly on the center line of the body, and the axial positioning cursor is at the level or slightly above the skeletal level. Enter the bed to the inner hole of the magnet after the locked position. All patients were selected to observe the L3-S1 segment and measure the diseased segment.

### 3.5. Main Observation Record Index

1. The facet joint angle value: the right facet joint angle is recorded as *X*, the left facet joint angle is recorded as *Y*, and the facet joint angle is recorded as *X* + *Y*.
2. The facet joint angle difference: the difference between the right facet joint angle *X* and the left facet joint angle *Y*, recorded as (*X* − *Y*), and the absolute value is recorded as *X* − *Y*.
3. Facet tropism (FT): it defines the absolute value of the difference between the angles of the left and right facet joints, namely, |*X* − *Y*|. |*X* − *Y*| > 10, as the facet joint is asymmetry.

### 3.6. Statistical Methods

Use Excel and SPSS20.0 software for data sorting and statistical analysis, and use pie chart, column chart, and line chart to display the results more intuitively. Count data are expressed by rate (%), using Pearson Chi-square test, grade data are expressed by rate (%), using rank sum test, multigroup comparison using Kruskal–Wallis *H* test, and *P* < 0.05 is used as the difference statistical learn meaning [20].

## 4. Experimental Results of Lumbar Disc Herniation

### 4.1. General Information Comparison

The study included 500 cases with an average age of 41.25 ± 3.02 years. There were 137 cases in the central LDH group, aged 20–60 years, 72 males and 65 females. There were 140 cases in the left paralateral LDH group, aged 19–60 years, with an average age of 41.17 ± 4.34 years and 75 males and 65 females. There were 127 cases in the right-side LDH group, aged 19–60 years, with an average age of 40.24 ± 1.25 years and 66 males and 50 females. There were 75 cases in the control group, aged 18–58 years old, with an average age of 40.34 ± 2.14 years and 35 males and 40 females. The age, gender, height, and weight of the four groups of cases included in the study were analyzed by variance analysis between groups, as shown in Table 1 and Figure 3. The difference was not statistically significant (*P* > 0.05). It means that comparisons between groups can be made. In addition, there was no statistically significant difference in age, *X*, *Y*, and *X* − *Y* between the men and women included in the study (*P* > 0.05).

### 4.2. Comparison of MRI and CT Measurement of Facet Joint Angle

Among the included cases, 115 cases underwent lumbar spine MRI examination and lumbar spine CT examination. Among them, there were 37 cases in the central LDH group, 40 cases in the left-side LDH group and 38 cases in the right-side LDH group. The *a* and *P* values of the L3/4, L4/5, and L5/S1 segment method measured by MRI and CT were subjected to independent sample *t* test, and the difference was not statistically significant (*P* > 0.05), as shown in Table 2 and Figure 4.

### 4.3. Comparison of the *T* and *P* Values of the L3/4, L4/5, and L5/S1 Segments of Each Experimental Group and the Control Group

The *a* and *P* values of the L3/4, L4/5, and L5/S1 segments of the central LDH group and the control group were compared by independent samples *t* test. The L4/5 and L5/S1 segments of the lesion in the central LDH group were significantly different from the *a* and *P* values of the same segment in the control group (*P* < 0.05); the adjacent segments were the same as the control group There was no significant difference in the *a* and *P* values of the segments (*P* > 0.05), as shown in Table 3 and Figure 5.

The *T* and *P* values of the L3/4, L4/5, and L5/S1 segments of the left-side LDH group and the control group were compared by independent samples *t* test. The L4/5 and L5/S1 segments of the left paralateral LDH group were significantly different from the *a* and *P* values of the same segment in the control group (*P* < 0.05), and the adjacent segment was compared with the control [21]. There was no significant difference in the *a* and *P* values of the same segment in the group (*P* > 0.05), as shown in Table 4 and Figure 6.

The *T* and *P* values of the L3/4, L4/5, and L5/S1 segments of the right lateral LDH group and the control group were compared by independent sample *t* test. The L4/5 and L5/S1 segments of the lesion in the right-side LDH group were significantly different from the *a* and *P* values of the same segment in the control group (*P* < 0.05). The adjacent segment was compared with the control. There was no statistically significant difference between the *a* and *P* values of the same segment in the group (*P* > 0.05), as shown in Table 5 and Figure 7.

## 5. Conclusion

This study summarizes the correlation between changes in the facet joint angle measured by MRI and lumbar disc herniation, but there are still shortcomings. In this study, each experimental group only included about 60–70 cases of lumbar disc herniation. Research on imaging measurement parameters, the subjectivity and error of the experimenter's data measurement, may affect the results of the experiment. The sample size included in the study is small, and the results have certain limitations, such as double-blind, multicenter, and large-sample randomized controlled studies, and the result will be more convincing. At the end of this study, the degree of facet joint and intervertebral disc degeneration was included in the research indicators. At the end, the experimental group of cases was stratified to study the differences in facet joint angles and asymmetry of different age groups, which are the shortcomings of this study. Clinically, the etiology of low back and leg pain is complicated and is not caused by a single factor. It is difficult to distinguish various factors when screening cases. Therefore, this study also has certain criteria for the diagnosis, inclusion, and exclusion of selected cases. This study is only a comparative study of morphological parameters and does not involve the research scope of biomechanics and etiology. MRI has high sensitivity for the measurement of the angle of the facet joints of the lumbar spine and can be used to study the correlation between the changes of the facet joint angles and the herniated disc. Facet joint asymmetry is closely related to lateral lumbar disc herniation, which may be one of its pathogenesis factors. The herniated intervertebral disc is mostly on the sagittal side of the facet joint, and the facet joint angle on the side of the herniated disc is more sagittal. The asymmetry of the facet joints is not related to the central lumbar disc herniation, and the angle of the facet joints on both sides of the central lumbar disc herniation is partial sagittal.

## Figures and Tables

**Figure 1:** Schematic of magnetic resonance imaging.

**Figure 2:** Interpretation of the shape of herniated intervertebral disc in MRI images.

**Figure 3:** Comparison of cases in each group.

**Figure 4:** Comparison of MRI and CT measurement of facet joint angle.

**Figure 5:** Comparison of *T* and *P* values between the central LDH group and the control group.

**Figure 6:** Comparison of *a* and *R* values between the left-side LDH group and the control group.

**Figure 7:** Comparison of *T* and *P* values between the right-side LDH group and the control group.

**Table 1:** Comparison of age, gender, height, and weight of cases in each group.

	Age	Gender		Height (cm)	Weight (kg)
		Male	Female		
Central LDH group	41.25 ± 3.02	72	65	162.28 ± 3.42	58.45 ± 3.31
Left-side LDH group	41.17 ± 4.34	75	65	163.42 ± 3.23	57.77 ± 5.35
LDH group on the right side	40.24 ± 1.25	66	50	162.91 ± 5.15	59.60 ± 4.72
Control group	40.34 ± 2.14	35	40	163.41 ± 4.25	59.42 ± 5.24
*F*	0.394	0.254		0.465	0.979
*P*	0.675	0.102		0.630	0.381

**Table 2:** Comparison of MRI and CT measurement of facet joint angle (unit: °).

	L3/4 segment		L4/5 segment		L5/S1 segment	
	*X*	*Y*	*X*	*Y*	*X*	*Y*
MRI	36.1 ± 4.8	36.3 ± 4.4	42.3 ± 5.1	43.7 ± 4.3	51.0 ± 3.6	43.4 ± 6.2
CT	36.6 ± 1.9	37.3 ± 5.4	42.4 ± 6.1	43.4 ± 5.1	50.5 ± 5.4	45.2 ± 5.5
*P*	0.442	0.721	0.425	0.753	0.325	0.521

**Table 3:** Comparison of *T* and *P* values between the central LDH group and the control group.

Segments		Comparison of control group and L4/5 central LDH		Comparison of control group and L5/S1 central LDH	
		*T*	*P*	*T*	*P*
L3/4 segment	*X*	−0.651	0.516	0.421	0.648
	*Y*	−0.608	0.544	0.603	0.565
L4/5 segment	*X*	−2.682	0.008^*∗*^	−0.621	0.536
	*Y*	−3.087	0.002^*∗*^	−1.061	0.290
L5/S1 segment	*X*	0.346	0.730	3.787	0.000^*∗*^
	*Y*	0.369	0.713	4.091	0.000^*∗*^

“^*∗*^” means that the difference between the two groups is significant.

**Table 4:** Comparison of *T* and *P* values between the left-side LDH group and the control group.

Segments	Comparison of control group and L4/5 left lateral LDH		Comparison between control group and L5/S1 left lateral LDH	
	*T*	*P*	*T*	*P*
L3/4 segment	−0.370	0.712	0.843	0.358
	−0.555	0.580	0.604	0.516
L4/5 segment	−3.093	0.000^*∗*^	−0.053	0.958
	3.235	0.002^*∗*^	−0.319	0.751
L5/S1 segment	0.348	0.728	−2.537	0.012^*∗*^
	0.401	0.689	3.113	0.000^*∗*^

“^*∗*^” means that the difference between the two groups is significant.

**Table 5:** Comparison of *T* and *P* values between the right-side LDH group and the control group.

Segments	Comparison between control group and L4/5 right lateral LDH		Comparison of control group and L5/S1 right lateral LDH	
	*T*	*P*	*T*	*P*
L3/4 segment	0.984	0.254	−0.546	0.831
	0.624	0.327	−0.275	0.376
L4/5 segment	3.319	0.534	−0.829	0.978
	−4.961	0.001^*∗*^	0.028	0.735
L5/S1 segment	−0.203	0.000^*∗*^	0.340	0.000^*∗*^
	−0.244	0.840	7.920	0.002^*∗*^

“^*∗*^” means that the difference between the two groups is significant.

## Data Availability

The data used to support the findings of this study are available from the corresponding author upon request.
